# The Effect Analysis of Carrier Gas Flow Rate on the Rapid Gas Chromatographic Separation System

**DOI:** 10.1155/2020/8886609

**Published:** 2020-11-06

**Authors:** Xu Zhang, Sixiang Zhang, Wei Zhou, Yang Qi

**Affiliations:** ^1^Tianjin Key Laboratory of High Speed Cutting and Precision Machining, School of Mechanical Engineering, Tianjin University of Technology and Education, Tianjin, China 300222; ^2^School of Mechanical Engineering, Hebei University of Technology, Tianjin, China 300100

## Abstract

Odor pollution did not only disturb the human normal life but also aroused the attention of environmental researchers and environmental protection departments. Therefore, the research on odor detecting method and instrument is important to theory and application. On this basis, the self-developed microfluidic chip capillary column is used in our odor detecting system. In this paper, lead the chip column into the chromatography separation system, with its small size, high efficiency, easy integration, and other characteristics to replace the original traditional column. The chip column was used in many gas experiments for several typical VOCs. At different carrier gas flow rates, the baseline value, toluene response, and toluene and methyl sulfide mixed gas separation were compared to verify the experiment to determine the optimal carrier gas flow rate in accordance with its response and separation degree. Under the premise of ensuring column efficiency as high as possible, it is determined that the optimal carrier gas flow rate is 6 ml/min. This paper shows the most proper carrier gas flow rate of our odor detecting system with the self-developed microfluidic chip capillary column.

## 1. Introduction

In recent years, industrial and agricultural production processes and household waste have emitted a large amount of volatile organic compounds (VOCs), causing a series of atmospheric pollution problems. VOCs cause harm to the human respiratory system, digestive system, and endocrine system. Common psychological and emotional injuries include irritability, dizziness, nausea, and vomiting. Environmental pollution has attracted the attention of all countries in the world. The environmental protection monitoring department not only wants to know where the pollution source is but also wants to know the type and concentration of pollutants. At present, the gas detection method at home and abroad is mainly gas chromatography. Chromatography technology is a general term for the separation of complex samples and is an important method for modern separation detection and analysis [1]. The traditional gas separation and detection equipment has a large volume and mass, the operation process is complex and time-consuming, the analysis speed is slow, and the separation gas mixture uses a longer column, resulting in a long analysis cycle. The research group developed and manufactured a chip-type column for this purpose. It has features such as small sample size, high detection efficiency, low use cost, portability, ease of integration with other technical equipment, and good compatibility [2]. The gas chromatography separation and detection system involved in this article uses Beijing Minnick's ten-way valve as the sample injection system, the chip-type column as the separation system, and the PID (Photoionization Detector) as the detection system. According to the rate theory, the carrier gas flow rate affects the column. Selecting the optimal carrier gas flow rate is of great significance for the evaluation of the instrument's performance and detection accuracy.

## 2. Experimental Part

### 2.1. Separation Principle of the Chip Column

The chip column uses the principle of separation by gas chromatography. In gas chromatography, the sample gas to be analyzed is rapidly carried by the carrier gas into the column. The column contains a solid or liquid stationary phase. The polarity, boiling point, or the physical and chemical properties of the adsorbed sample are different. As a result, the components are constantly distributed or adsorbed/desorbed between the stationary phase and fluidity, resulting in different rates of the components flowing out of the column, so that the retention time of the components in the column is different, in chronological order flow out of the column and into the end of the detector for detection [3].

### 2.2. Processing of the Chip Column

The chip column utilizes the fine sandblasting jet process to etch the surface of the borosilicate glass and adopts an anodic bonding processing method to process a Pyrex type borosilicate glass material chip with a size of 115 mm × 60 mm × 6 mm as shown in Figure 1. The channel is designed as an S-channel with a circular cross section, which has the advantage of ensuring that the gas molecules of the components travel the same path inside and outside the chip column channel with the same column volume [4]. The channel has an inner diameter of 400 *μ*m and a length of 5.8 m. In order to achieve the separation of VOCs, three kinds of fixing solutions, 100% dimethylpolysiloxane, 14% cyanopropylphenyl-86% dimethylpolysiloxane, and polyethylene glycol, were, respectively, applied. The pipe connection method of the chip is connected by means of a clamp fixture and is connected by a PTFE pipe with a threaded connection, and the connection head is connected by a conical pressure ring and can withstand a temperature of 300°C.

## 3. Chromatographic Rate Theory

### 3.1. Several Parameters for Evaluating Column Performance

The theoretical plate number *N* and the theoretical plate height *H* are the two main indicators reflecting the column performance of the column [5]. The calculation formula of *N* is

(1) $$\begin{array}{c} N=5.54{\left(\frac{t_{R}}{W_{1/2}}\right)}^{2}=16{\left(\frac{t_{R}}{W_{b}}\right)}^{2}, \end{array}$$

where *t*_*R*_ is the retention time, which refers to the time from the start of sampling until the sample passes the column to produce the highest peak; *W*_*b*_ is the width of the bottom of the peak, which refers to the tangent line at the inflection point of the chromatographic peak outflow curve. The distance between the base of the peak or the base line intersecting two points, *W*_1/2_, is the half width of the peak, which refers to the distance between the line parallel to the base of the peak at the midpoint of the peak height and the point of intersection on both sides of the peak [6].

*H*'s formula is

(2) $$\begin{array}{c} H=\frac{L}{N}, \end{array}$$

where *L* is the length of the column.

It can be seen that the narrowing of the chromatographic peaks and the height of the trays will increase the column efficiency. *N* and *H* are the main indicators that describe the performance of a column.

The degree of separation of components—the degree of separation [7] is calculated as

(3) $$\begin{array}{c} R=\frac{2\left(t_{R2}-t_{R1}\right)}{Y_{1}+Y_{2}}, \end{array}$$

where *Y*_1_, *Y*_2_ is the peak width of the peak.

The size of *R* can quantitatively reflect the degree of separation between components. When the chromatographic peak shape is asymmetrical or there is a slight overlap between adjacent two peaks, it is difficult to measure the peak width at the bottom. Instead, half width can be used instead. At this time, the resolution *R* can be expressed as

(4) $$\begin{array}{c} R=\frac{1.18\left(t_{R2}-t_{R1}\right)}{Y_{1/2\left(1\right)}+Y_{1/2\left(2\right)}}, \end{array}$$

where *Y*_1/2(1)_, *Y*_1/2(2)_ is the peak width at the half height of the peak.

### 3.2. Rate Theory

The column efficiency is the highest when the column and the sample are at a certain flow rate [8], and the relationship of *H*‐*u* is

(5) $$\begin{array}{c} H=A+\frac{B}{u}+Cu, \end{array}$$

where *H* is the tray height, *u* is the carrier gas velocity, and *A*, *B*, and *C* are three constants, where *A* is the eddy diffusion term, *B* is the molecular diffusion coefficient, and *C* is the mass transfer resistance factor. Equation (5) is a simplified version of the Van Deemter equation. According to equation (5), the height *H* of the tray measured at different flow rates is plotted against the flow rate *u* to obtain the *H*‐*u* curve, as shown in Figure 2. At the lowest point of the *H*‐*u* curve, the height of the theoretical plate *H* is the smallest, and the efficiency of the column is the highest. The flow rate corresponding to this point is the best flow rate *u*_best_. *H*_min_ and *u*_best_ can be differentiated by equation (5). Seek, that is,

(6) $$\begin{array}{c} \frac{dH}{\;du}=-\frac{B}{u^{2}}+C=0, \end{array}$$

(7) $$\begin{array}{c} u_{\text{best}}=\sqrt{\frac{B}{C}}. \end{array}$$

Bring formula (6) into formula (5):

(8) $$\begin{array}{c} \;H_{\min}=A+2\sqrt{BC}. \end{array}$$

In actual work, try to shorten the analysis time without significantly affecting the efficiency of the column. The flow rate is usually slightly higher than the optimal flow rate.

The relationship of the constant terms *A*, *B*, and *C* is brought into equation (5).

(9) $$\begin{array}{c} H=2\lambda d_{p}+\frac{2\gamma D_{g}}{\mu }+\left[\frac{0.01k^{2}}{{\left(1+k\right)}^{2}}∙\frac{d_{p}^{2}}{D_{\text{g}}}+\frac{2}{3}\cdot \frac{k}{{\left(1+k\right)}^{2}}∙\frac{d_{f}^{2}}{D_{1}}\right]\mu . \end{array}$$

According to equation (9), the column packing uniformity, carrier particle size, carrier gas type, carrier gas flow rate, column temperature, and liquid film thickness of the stationary phase have effects on column efficiency and peak expansion.

## 4. Experiments and Data

### 4.1. Experimental Device and Conditions

In order to understand the effect of carrier gas flow on separation of mixtures, the self-developed odor detecting online system is introduced in these experiments. The system is shown in Figure 3.

There are six units in the system, including the gas channel unit, injection unit, separating unit, detecting unit, controlling unit, and data processing unit. This system has passed the stability testing, systematic linearity testing, and sensitivity testing. The testing experiments show that the baseline fluctuation value is less than 2.3 mV; the linearity of the system for xylene, ethanol, and butane is 99.98%, 99.99%, and 99.98%, respectively. The sensitivity was 1 ppm, 0.8 ppm, and 0.6 ppm, respectively [9]. We will not elaborate the testing experiments of our self-developed odor detecting online system.

The following experiment is done under the normal operating conditions. The normal operating conditions are as follows: (1) 99.999% nitrogen (N_2_) was used as carrier gas; (2) the lab environmental temperature is at 25°C; (3) the pressure in the laboratory is 0.101 MPa.

### 4.2. Effect of Carrier Gas Flow on Baseline Value

Baseline refers to the signal curve produced by the detector when only nitrogen passes through the column and detector under normal operating conditions. The ideal stable baseline should be a horizontal straight line. The peak height is the vertical distance between the highest point of the chromatographic peak and the bottom of the peak and the vertical distance between the highest point of the chromatographic peak and the baseline. In gas chromatography, the peak height is one of the commonly used quantitative parameters. From the theory of velocity, the flow affects the height of the theoretical plate, thus affecting the size of the baseline value. By changing the flow rate before the column, the voltage value of the PID is monitored with a voltmeter. After the baseline is stabilized, the corresponding baseline value is obtained. We used 99.999% nitrogen (N_2_) as carrier gas in this experiment. The carrier gas flow rate changed from 0 ml/min to 9 ml/min at 25°C in the lab. The effect of carrier gas flow on baseline values is shown in Figure 4. It shows that the baseline value was low while the carrier gas flow speeded up.

### 4.3. Effect of Carrier Gas Flow Rate on Toluene Response

From the rate theory, the flow rate of the carrier gas has an opposite effect on the mass transfer resistance term and the vertical diffusion term. If the carrier gas velocity *u* increases, the longitudinal diffusion term decreases so that the column efficiency increases, but at the same time, the mass transfer resistance term increases, which in turn reduces the column efficiency. The flow rate of the carrier gas influences the height of the tray, so there is an optimum flow rate so that the column efficiency is the highest. In this experiment, the sample gas was sampled using 200 ppb toluene standard gas prepared by DaLian Date and the carrier gas used was 99.999% nitrogen (N_2_). By changing the flow rate of the carrier gas before the column, the corresponding response value of the 200 ppb toluene standard gas is shown in Figure 5. It shows that toluene response value had a peak value at about 6 ml/min.

### 4.4. Effect of Carrier Gas Flow on Separation of Mixtures

A gas generator was used to prepare dimethyl sulfide and toluene gas mixture. The gas mixture was separated and detected by the gas chromatographic separation and detection system developed by our group [10, 11]. In this experiment, 99.999% nitrogen (N_2_) was used as the carrier gas. The temperature of the chip column is 85°C, select the S48 300/HMT type mass flow controller manufactured, and control the flow rate at 2~7 ml/min, and each flow rate is carried out. Two repeated injection tests were performed to determine the retention time and peak width of the mixture, and the mean value was calculated. Separation of the mixture is mainly achieved by using the separation of the system; the relative physical and chemical properties such as the boiling point, polarity, and adsorption and desorption of each component are fixed [12]. After separation and detection of dimethyl sulfide and toluene mixture, data processing was performed using the software of the upper computer to calculate the retention time and peak width of dimethyl sulfide and toluene at different flow rates, and the separation was calculated according to equation (3). The specific data results are shown in Table 1.

From Table 1, the flow rate is between 2 and 7 ml/min, the separation degree of methyl sulfide and toluene is *R* > 1.5, and the two peaks are completely separated. The higher the degree of separation, the more accurate detection results could be [13]. When the flow rate is low, as the flow rate increases, the peak width of the peak narrows, the retention time becomes shorter, the number of theoretical plates becomes larger, and the column efficiency of the chip column increases [14].

## 5. Conclusions

During the rate theory, the flow rate of the carrier gas affects the column and column efficiency. Using the developed chip-type column at different carrier gas flow rates, experiments were carried out to examine the effect of carrier gas flow rate on the baseline value, 200 ppb toluene response, and mixture separation. The flow rate was between 2 and 7 ml/min, and the baseline value gradually decreased. The response value of 200 ppb toluene reached maximum at a flow rate of about 6 ml/min. The separation of dimethyl sulfide and toluene was not less than 1.5. Both were completely separated. Based on comprehensive column efficiency, gas response value, high separation of mixed gas, short analysis cycle, and other factors, the optimal carrier gas flow rate for the chip column is 6 ml/min.

## Figures and Tables

**Figure 1:** The self-developed microfluidic chip capillary column.

**Figure 2:** Relation curve between plate height and the carrier gas line speed.

**Figure 3:** Self-developed odor detecting online system.

**Figure 4:** Effect of carrier gas flow rate on the baseline value.

**Figure 5:** Effect of carrier gas flow rate on 200 ppb toluene response value.

**Table 1:** Dimethyl sulfide and toluene separation results in different carrier gas flow rates.

Flow rate (ml/min)	Substance category	Retention time (s)	Peak width	Separation degree
2	Dimethyl sulfide	78	26	2.79
	Toluene	176	44	
2.5	Dimethyl sulfide	65	37	2.13
	Toluene	146	39	
3	Dimethyl sulfide	55	46	1.66
	Toluene	127	41	
3.5	Dimethyl sulfide	47	46	1.51
	Toluene	107	34	
4	Dimethyl sulfide	44	33	1.68
	Toluene	96	29	
4.5	Dimethyl sulfide	37	33	1.53
	Toluene	85	29	
5	Dimethyl sulfide	34	26	1.68
	Toluene	76	24	
5.5	Dimethyl sulfide	28	20	1.63
	Toluene	61	21	
6	Dimethyl sulfide	26	26	1.50
	Toluene	60	20	
6.5	Dimethyl sulfide	24	20	1.74
	Toluene	57	18	
7	Dimethyl sulfide	23	23	1.58
	Toluene	54	16	

## Data Availability

The data used to support the findings of this study are included within the article.
